# Long Noncoding RNA KIAA0125 Potentiates Cell Migration and Invasion in Gallbladder Cancer

This article has been retracted.

**DOI:** 10.1155/2015/108458

**Published:** 2015-09-13

**Authors:** Wenjie Lv, Lei Wang, Jianhua Lu, Jiasheng Mu, Yingbin Liu, Ping Dong

**Affiliations:** Department of General Surgery, Xinhua Hospital Affiliated to School of Medicine, Shanghai Jiao Tong University, 1665 Kongjiang Road, Shanghai 200092, China

## Abstract

Gallbladder cancer (GBC) is one of the mostly aggressive diseases with poor prognosis due to the lack of severe symptoms. To date, little is known about the potential roles and underlying mechanisms of long noncoding RNAs (lncRNAs) in GBC initiation and progression. Thus, it provides us with a novel insight into the contribution of lncRNAs to GBC development. Remarkably, we found the differential expression of a lncRNA, namely, KIAA0125, in a pair of GBC cell sublines which possess different metastatic potentials. Then the effects of KIAA0125 on GBC cell migration, invasion, and epithelial-mesenchymal transitions (EMT) were investigated by using a lentivirus-mediated RNA interference (RNAi) system. Notably, cell migration and invasion were strongly inhibited by KIAA0125 suppression. Moreover, the expression of *β*-Catenin was increased and the expression of Vimentin was decreased in GBC-SD/M cells after KIAA0125 knockdown. Thus, our findings suggested that KIAA0125 promoted the migration and invasion of GBC cells and could serve as a potential therapeutic target in advanced GBC.

## 1. Introduction

Gallbladder cancer (GBC) is one of the most lethal malignancies and the fifth common neoplasm of gastrointestinal tract [1–3]. The 5-year survival rate is extremely low, possibly due to the lack of severe symptoms and thus it is hard to make a diagnosis at an early stage [4]. Moreover, treatment approaches such as cholecystectomy, chemotherapy, or radiotherapy in advanced cases did not yield favorable outcomes [4–8]. Hence, exploring novel signal molecules involved in GBC metastasis may provide new effective therapeutic strategies.

Recently, an increasing number of investigations have shown that long noncoding RNAs (lncRNAs), a group of newly identified noncoding RNA molecules, are emerging as key players in the regulation of multiple stages of many cancers, such as colorectal cancers, prostate cancer, hepatocellular carcinomas, and breast cancers [9–15]. For instance, the aberrant expression of Hox transcript antisense intergenic RNA (HOTAIR) has been identified in some cancers, which has been shown to correlate with cellular proliferation, metastasis, and clinical relapse [10, 16, 17]. The human metastasis associated lung adenocarcinoma transcript 1 (MALAT-1) is known to be misregulated in several cancers and usually acts as a critical regulator of cancer metastasis and epithelial-mesenchymal transitions (EMT) [18–20]. Yet, it is still obscure whether lncRNAs are involved in GBC progression.

Intriguingly, a novel lncRNA, namely, KIAA0125, draws our attention. The* KIAA0125 *gene is localized on chromosome 14q32.33. A recent study reported that* KIAA0125 *might play a role in neurogenesis, maybe in preventing the generation of dopaminergic neurons, or it could also be involved in inducing astrocytosis. However, the functional role of KIAA0125 in cancer has not been determined yet. In the present study, we investigated whether KIAA0125 is involved in GBC progression. We found KIAA0125 expression is incredibly elevated in a GBC cell subline GBC-SD/M with higher metastatic potentials as compared to the other subline GBC-SD cells [21]. A lentivirus-mediated RNA interference (RNAi) system was thus employed to knock down KIAA0125 expression in GBC-SD/M cells. Moreover, the effects of KIAA0125 on GBC cell migration and invasion were further evaluated.

## 2. Materials and Methods

### 2.1. Cell Culture

Two human GBC cell sublines, GBC-SD and GBC-SD/M, which possess lower and higher metastatic potential, respectively [21], were obtained from the Type Culture Collection of the Chinese Academy of Sciences (Shanghai, China). The two cell sublines were cultured in DMEM (# 11995065; Gibco Life Technology, Gaithersburg, MD) supplemented with 10% fetal bovine serum (FBS; Biowest, Nuaille, France). HEK293T cells were grown in DMEM (# SH30243.01B+; HyClone, Logan, Utah, USA) containing 10% FBS. All cells were grown at 37°C in an incubator with 5% CO_2_.

### 2.2. Lentivirus Construction

An shRNA sequence (5′-GCAAGGCCAGTGGAGTTAATCCTCGAGGATTAACTCCACTGGCCTTGC-3′) was designed based on human lncRNA gene KIAA0125 (NR_026800). The nontargeting shRNA (5′-GCGGAGGGTTTGAAAGAATATCTCGAGATATTCTTTCAAACCCTCCGCTTTTTT-3′) was used as control. Then two shRNA sequences were cloned into pFH-L vectors (Shanghai Hollybio, China), which contain green fluorescent protein (GFP) as the detectable marker. The two reconstructed vectors were then transfected into HEK293T cells to generate lentiviruses, along with pCMVΔR8.92 and pVSVG-I as packing vectors (Shanghai Hollybio, China). Supernatants containing either the lentivirus expressing the KIAA0125 shRNA (Lv-shKIAA0125) or the control shRNA (Lv-shCon) were harvested 96 h after transfection.

### 2.3. Lentivirus Infection

GBC-SD/M cells were applied for KIAA0125 knockdown, which were cultured in 6-well plates at a density of 5 × 10^4^ cells/well. Then GBC-SD/M cells were subjected to Lv-shKIAA0125 and Lv-shCon treatment for 96 h, with a multiplicity of infection (MOI) of 50. To evaluate the infection efficiency, cells were observed under fluorescence microscope and the percentage of GFP positive cells was counted.

### 2.4. Quantitative Real-Time PCR

Total RNA was extracted from GBC-SD/M cells using the Trizol reagent (Invitrogen, Carlsbad, CA, USA). For each sample, 2 *μ*g of total RNA was subjected to reverse transcription by using Mu-MLV (MBI Fermentas, Euromedex, Souffelweyersheim, France). Then the expression levels of four candidate genes (KIAA0125, *α*-Catenin, *β*-Catenin, and Vimentin) in each cDNA sample were analyzed using primers listed below. Beta-actin and GAPDH were used as internal control genes. For each 20 *μ*L PCR reaction, we added SYBR Premix Ex Taq (10 *μ*L), forward and reverse primers (2.5 *μ*M, 0.8 *μ*L), cDNA sample (5 *μ*L), and ddH_2_O (4.2 *μ*L). The Bio-Rad Connect real-time PCR platform was applied to run PCR reactions for 40 cycles under the following conditions: (1) initial denaturation at 95°C for 1 min, (2) denaturation at 95°C for 5 s, and (3) annealing extension at 60°C for 20 s. Mathematical model for relative quantification in real-time PCR was 2^−ΔΔCT^ method [22]. Data were presented as CT values, which were defined as the threshold PCR cycle number at which an amplified product is first detected: ΔCT = Avg. CT (target gene) – Avg. CT (housekeeping gene), and ΔΔCT = Avg. ΔCT − Avg. ΔCT (control). Results presented in histogram are the normalized target gene amount relative to control 2^−ΔΔCT^. Primers are listed as follows:

 KIAA0125 (*KIAA0125*, ID: 9834):
 5′-CCTCTCAGCCTCCAGCGTTG-3′ (forward)
 5′-TGCTCTTGCTCACTCACACTCC-3′ (reverse)
 Vimentin (*VIM*, ID: 7431):
 5′-ATTCCACTTTGCGTTCAAGG-3′ (forward)
 5′-CTTCAGAGAGAGGAAGCCGA-3′ (reverse)
 
*α*-Catenin (*CTNNA1*, ID: 1495):
 5′-GAGCTGTCTACGCAAGTCCC-3′ (forward)
 5′-TTTCGGAGTACATGGGCAAT-3′ (reverse)
 
*β*-Catenin (*CTNNB1*, ID: 1499):
 5′-AGCTACTGCCTCCGGTCTTC-3′ (forward)
 5′-GTGGTCAACAGCCAGCTCA-3′ (reverse)
 
*β*-actin (*ACTB*, ID: 60):
 5′-GTGGACATCCGCAAAGAC-3′ (forward)
 5′-AAAGGGTGTAACGCAACTA-3′ (reverse)
 GAPDH (*GAPDH*, ID: 2597):
 5′-GGAAGCTTGTCATCAATGGAA-3′ (forward)
 5′-TGGACTCCACGACGTACTCA-3′ (reverse).

### 2.5. The Scratch Test

Random migration was determined by the scratch test assay, in which cells were grown to 90% confluency in 96-well plates, streaked with a 200 *μ*L sterile pipette tip, and allowed to recover in an incubator at 37°C in the next 36 h. The plates were visualized under light microscope and fluorescence microscope (×40 magnification) at 24 h and 36 h. Random migration was evaluated by measuring the area of occupancy via an image-analysis program (Image-Pro Plus, Media Cybernetics, MD).

### 2.6. Transwell Assay

Transwell chambers and Matrigel Invasion Chambers (Corning, NY, USA) were used for transwell assay and transwell invasion assay, respectively. For transwell assay, cells were harvested and suspended in serum-free medium. Then 200 *μ*L cell suspension was added to the upper chamber at a density of 3 × 10^4^ cells/well, and 500 *μ*L of serum-rich medium was added to the lower chamber. The transwell chambers were cultured for 6 h. For transwell invasion assay, the Matrigel Invasion Chambers were incubated for 16 h. In both analyses, the chambers were collected for the following treatment. The surface of the upper chamber was swabbed with cotton-tipped applicators to remove the cells that did not migrate. The lower compartment was fixed with methanol and stained by crystal violet. Distilled water was then applied to wash off excess stain materials. For data analysis, migrating cells and the amount of dissolved crystal violet were both measured by using a light microscope and spectrophotometer.

### 2.7. Statistical Analysis

All assays were performed in triplicate and the data were expressed as mean ± standard deviation (SD). The Student's *t*-test was applied for statistical analysis and a *P* value of less than 0.05 was considered significant.

## 3. Results

### 3.1. Suppression of KIAA0125 by Lentivirus-Mediated RNAi

Here we firstly detected the expression of KIAA0125 in human GBC-SD and GBC-SD/M cells using qRT-PCR analysis. As shown in Figure 1, the relative expression level of KIAA0125 was remarkably upregulated in GBC-SD/M cells (5.85 ± 0.357), compared to GBC-SD cells (1.003 ± 0.087). As previously described by Liu and his colleagues, GBC-SD and GBC-SD/M had relative lower and higher metastatic potential, respectively. The GBC-SD/M subline was established by isolating a subpopulation with high metastatic potential from an experimental liver metastatic model of GBC [21]. Hence, our data strongly suggest that KIAA0125 is involved in the regulation of GBC metastasis. To verify the role of KIAA0125 in GBC, we employed a lentivirus-mediated RNAi system to specifically knock down the expression of KIAA0125 in GBC-SD/M cells. Our constructed lentiviruses could successfully infect GBC-SD/M cells, with an infection efficiency more than 80% (Figure 2(a)). The relative expression level of KIAA0125 in Lv-shKIAA0125 infected cells was much lower than in Lv-shCon infected cells, with a knockdown efficiency more than 60% (Figure 2(b)). These results indicated that Lv-shKIAA0125 could specifically knock down KIAA0125 in GBC-SD/M cells.

### 3.2. Suppression of KIAA0125 Inhibited GBC Cell Migration

To testify our hypothesis that KIAA0125 may contribute to GBC migration, we performed the scratch test and transwell assay in GBC-SD/M cells treated with Lv-shKIAA0125. Compared with Lv-shCon group, the “wound healing” ability of Lv-shKIAA0125 treated cells was significantly inhibited as shown by the reduced areas of occupancy at indicated time points (Figures 3(a) and 3(b)). Moreover, we observed remarkable reduction of cells that migrated to the lower compartment in Lv-shKIAA0125 group (Figure 4(a)). The number of migrating cells was reduced in Lv-shKIAA0125 group by 67%, as compared to Lv-shCon group (Figure 4(b)). The amount of crystal violet was also decreased by 55% after KIAA0125 suppression (*P* < 0.001, Figure 4(c)). However, the impact of KIAA0125 knockdown on GBC-SD cell migration was negligible, as determined by transwell assay (Figure S1(A) in Supplementary Material available online at http://dx.doi.org/10.1155/2015/108458). As shown in Figure S1(B), the number of migrating cells was reduced in Lv-shKIAA0125 group by 29%, as compared to Lv-shCon group. Also, the amount of crystal violet was decreased by only 7% (Figure S1(C)). These results strongly indicate that KIAA0125 is a key regulator of GBC cell motility and migration.

### 3.3. Suppression of KIAA0125 Inhibited GBC Cell Invasion

Furthermore, the invasive potential of Lv-shKIAA0125 treated cells was evaluated by transwell assay using Matrigel Invasion Chambers. As shown in Figures 5(a) and 5(b), the number of cells that invaded to the lower compartment was markedly reduced after KIAA0125 suppression (164.9 ± 6.5), as compared to Lv-shCon group (205.9 ± 2.4), which was confirmed by the amount of crystal violet (Figure 5(c)). These results indicate that KIAA0125 also facilitates GBC cell invasion.

### 3.4. Effect of KIAA0125 Suppression on EMT

To determine the underlying molecular mechanism by which KIAA0125 controls GBC metastasis, we analyzed the effect of KIAA0125 knockdown on EMT, which has been shown to play a key role in promoting the aggressiveness of GBC [23]. Three EMT markers, Vimentin, *α*-Catenin, and *β*-Catenin, were selected for qRT-PCR analysis. As shown in Figure 6, the relative expression level of Vimentin in Lv-shKIAA0125 infected cells was much lower than in Lv-shCon infected cells, with a reduction by over 10%. The relative expression level of *β*-Catenin was remarkably elevated by about 40% after KIAA0125 knockdown. However, the expression of *α*-Catenin was not significantly changed. Our data suggest that KIAA0125 is essential for GBC metastasis possibly due to the induction of EMT.

## 4. Discussion

LncRNAs can be classified into several subtypes including intergenic, intronic, sense, antisense, and bidirectional according to their genomic relationship with coding genes [24, 25]. In the present study, we found a differentially expressed lncRNA named KIAA0125 in GBC-SD and GBC-SD/M using qRT-PCR analysis. KIAA0125 was upregulated in a highly metastatic GBC cell subline GBC-SD/M, in contrast to GBC-SD cell subline with a relative lower metastatic potential. More importantly,* in vitro* studies revealed that knockdown of KIAA0125 had an inhibitory effect on GBC cell motility, migration, and invasion. So far, little is known about the biological roles of lncRNAs in GBC initiation and progression, even though many of them are known to be misregulated in various cancer types and involved as a key regulator during carcinogenesis [10, 16–20]. Hence, the present study presents us with a novel insight into the contribution of lncRNAs in GBC metastasis.

EMT, originally viewed as a phenotype switch in developmental biology, has been linked to carcinoma invasion and metastasis in recent years. EMT can be recognized as a manifestation of extreme epithelial cell plasticity, which involves derangement of apicobasal polarity, regulation of cell-to-cell adhesive architecture, loss of basal lamina integrity, and lack of cell shape plasticity [26, 27]. In many circumstances, EMT leads to increased translocation (migration) ability and participates in cancer metastasis [28–30]. In GBC, EMT also plays an important role in promoting the aggressiveness of cancer cells [4]. A great number of molecules change in expression and distribution during the EMT, including Catenins, Cadherins, Vimentin, and integrins [31]. Remarkably, we observed that after KIAA0125 knockdown, the expression of Vimentin was downregulated and the expression of *β*-Catenin was upregulated. Vimentin, a major component of the intermediate filament family, is known to maintain cellular integrity and thus its overexpression may result in accelerated cell growth, invasion, and poor prognosis in many cancers [32]. *β*-Catenin is typically more abundant in epithelial-like cells, and loss of *β*-Catenin is a hallmark of EMT [33]. Taken together, we may infer that KIAA0125 promotes GBC cell migration and invasion partly via induction of Vimentin and suppression of *β*-Catenin. However, further investigation is needed to clarify the sophisticated regulatory mechanism underlying this process.

In all, we described for the first time the function of KIAA0125 in GBC cell migration, invasion, and EMT. Our findings suggest that KIAA0125 may serve as a potential therapeutic target for advanced GBC cases. More detailed research would be crucial to evaluate the biological function of KIAA0125 in tumor samples from GBC cases.

## Supplementary Material

Figure S1: Effect of KIAA0125 knockdown on cell migration in GBC-SD cells. (A) Cells migrated to the lower chamber was stained by crystal violet and photographed. Scale bar: 100 µm. (B) The number of migrated cells and (C) the amount of crystal violet in both groups were measured. ^*^P<0.05, compared to Lv-shCon.

## Figures and Tables

**Figure 1:** KIAA0125 expression in human GBC cells. The mRNA expression levels of KIAA0125 in GBC-SD and GBC-SD/M cells were determined by qRT-PCR. *β*-Actin was used as an internal control gene. ^***^ *P* < 0.001, compared to GBC-SD.

**Figure 2:** Knockdown of KIAA0125 by lentivirus-mediated RNAi. (a) GBC-SD/M cells were infected with Lv-shKIAA0125 or Lv-shCon, and the infection efficiency was monitored by fluorescence microscopy after 96 h. Scale bar: 100 *μ*m. (b) The knockdown efficiency of KIAA0125 targeting lentivirus-mediated RNAi was determined by qRT-PCR. *β*-Actin and GAPDH were used as internal control genes. ^***^ *P* < 0.001, compared to Lv-shCon.

**Figure 3:** Effect of KIAA0125 knockdown on wound healing. (a, b) The wound healing ability of GBC-SD/M cells was evaluated by using the scratch test after Lv-shKIAA0125 or Lv-shCon treatment at 24 h and 36 h after wound. Scale bar: 250 *μ*m. ^*^ *P* < 0.05, compared to Lv-shCon.

**Figure 4:** Effect of KIAA0125 knockdown on cell migration. The migration of Lv-shKIAA0125 or Lv-shCon treated cells was evaluated using the transwell assay. (a) Cells migrating to the lower chamber were stained by crystal violet and photographed. Scale bar: 100 *μ*m. (b) The number of migrating cells and (c) the amount of crystal violet in both groups were measured. ^**^ *P* < 0.01, ^***^ *P* < 0.001, compared to Lv-shCon.

**Figure 5:** Effect of KIAA0125 knockdown on cell invasion. The invasive ability of Lv-shKIAA0125 or Lv-shCon treated cells was evaluated using the Matrigel Invasion Chambers. (a) Cells invading to the lower chamber were stained by crystal violet and photographed. Scale bar: 100 *μ*m. (b) The number of migrating cells and (c) the amount of crystal violet in both groups were measured. ^*^ *P* < 0.05, ^**^ *P* < 0.01, compared to Lv-shCon.

**Figure 6:** Effect of KIAA0125 knockdown on EMT. The mRNA expression levels of molecules (Vimentin, *α*-Catenin, and *β*-Catenin) involved in EMT was examined in Lv-shKIAA0125 or Lv-shCon treated groups. *β*-Actin and GAPDH were used as internal control genes. ^*^ *P* < 0.05, ^**^ *P* < 0.01, compared to Lv-shCon.
